This article has been retracted.

# A freight integer linear programming model under fog computing and its application in the optimization of vehicle networking deployment

**DOI:** 10.1371/journal.pone.0239628

**Published:** 2020-09-24

**Authors:** Xiaowen Wang, Peng Qiu

**Affiliations:** 1 China Academy of Transportation Sciences, Beijing, China; 2 China Academy of Railway Sciences Corporation, Beijing, China; University College London, UNITED KINGDOM

## Abstract

The increase in data amount makes the traditional Internet of Vehicles (IoV) fail to meet users’ needs. Hence, the IoV is explored in series. To study the construction of freight integer linear programming (ILP) model based on fog computing (FG), and to analyze the application of the model in the optimization of the networking deployment (ND) of the IoV. FG and ILP are combined to build a freight computing ILP model. The model is used to analyze the application of ND optimization in the IoV system through simulations. The results show that while analyzing the ND results in different scenarios, the model is more suitable for small-scale scenarios and can optimize the objective function; however, its utilization rate is low in large-scale scenarios. While comparing and analyzing the network cost and running time, compared with traditional cloud computing solutions, the ND solution based on FG requires less cost, shorter running time, and has apparent effectiveness and efficiency. Therefore, it is found that the FG-based model has low cost, short running time, and apparent efficiency, which provides an experimental basis for the application of the later deployment of freight vehicles (FVs) in the Internet of Things (IoT) system for ND optimization. The results will provide important theoretical support for the overall deployment of IoV.

## 1. Introduction

With the rapid development of science and technology, the living standards of humans are constantly improving. Meanwhile, the process of urbanization is accelerating, and the construction of urban agglomerations (UAs) has received wide attention. However, with the increase in the scale of UAs, many people and economic activities have gathered to the larger UAs, making their breadth and intensity continue to increase. Consequently, inconsistent socio-economic development occurs, such as the continuous expansion of urban land occupation, the low utilization rate of lands, the rapid resource consumption, the limited environmental carrying capacity, and inadequate access to public services of residents. These are all examples of uncoordinated development [1, 2]. The emergence of these contradictions has seriously affected the balanced development of UAs. To resolve these contradictions, researchers and scholars have paid their attention to urban development. Lv et al. (2019) designed an environment monitoring system for smart cities based on the ZigBee wireless network; this system employed street lights as routes and taxis as nodes; after the network was dynamically organized, an address was assigned to each node as a unique identifier in the network [3]. This accomplishment shows that IoV is an essential research step in the research of smart cities.

The imbalanced development of UAs is often solved through the links between cities. The degree of closeness between cities is often reflected in two aspects. One is the flow of goods and people between cities. The flow of demand for goods reflects not only the population and infrastructure density in the area but also the fluctuations in productivity in this city. Therefore, freight data are utilized to effectively characterize the transportation relationship between cities or regions [4]. Generally, freight data include data on roads, railways, waterways, and aviation, among which road transportation has the characteristics of medium and short-distance transportation and a wide range of applications, accounting for more than 70% of the total freight amount [5]. Freight transportation is a part of transportation; thus, it is critical to extract the information about its real-time status. With the application of big data, Internet of Things (IoT), cloud computing, and other technologies, various mobile devices and sensors are connected to the network, generating huge amount of data [6]. Freight vehicles (FVs) are also equipped with various mobile communication devices, which are connected to the network during driving, thereby generating massive data. These big data are transmitted to the core network through receiving and processing. However, as the amount of data continues to increase, the core network has a blockage. In real life, once the data center fails, or a problem occurs in any section from the terminal to the core network and platform, it may cause huge security risks. Therefore, the real-time and security requirements on big data are extremely high [7]. As the socialization process accelerates, to reduce the analysis pressure of cloud computing and slow down the increase in transmission rate and delay of data, fog computing (FG) is proposed. It is a new technology that collects, processes, and analyzes data through the edge of the network, providing a powerful support for the Internet of Vehicles (IoV). Besides, its application has advantages [8]. Fog computing has several distinct features: low latency, location awareness, wide geographic distribution, mobile applications, and more edge nodes. These features make the deployment of mobile services more convenient, satisfying a wider range of node access. Compared to cloud computing, the architecture adopted by fog computing is more distributed and closer to the network’s edge. Fog computing concentrates data, data processing, and applications in devices at the edge of the network instead of storing almost all of them in clouds as cloud computing does.

In summary, for the emergence of massive data and the rapid growth of FVs, the traditional vehicle network system has weak data processing capabilities, which cannot meet the needs of many users on the network access. Therefore, to optimize the deployment of the IoV, this study combines FG and integer linear programming (ILP) to build a FG-based freight ILP model, explore its application for networking deployment (ND) optimization in the IoV system, and simulate its applications, thereby providing new ideas for the future application of FVs in ND and optimization under the IoT.

## 2. Literature review

With the rapid development of science and technology, researches on the IoV are constantly increasing. Meanwhile, FVs are the most common type of vehicles. The real-time extraction of their data and understanding of their trips have also been explored by many scholars. Le Pira et al. (2017) combined discrete choice models (DCMs) and agent-based models (ABMs) to plan urban freight transportation (UFT) network data; finally, the added values of UFT decision were proved [9]. To improve the transportation performance of the freight industry, Keya et al. (2018) proposed a mixed utility-regret-based mode selection model and set up a scenario for simulation. The results showed that the introduction of automation in the freight industry was more beneficial to the long-distance rental truck mode than the short-distance private truck mode; besides, as the transportation route and time increased, the mode shift was also critical [10]. Based on the travel data of FVs, Zhang et al. (2019) used a complex network method to describe cargo transportation from a multidimensional perspective; also, based on network analysis indicators of complex network theory, the topology and complexity of the freight network were performed. The results showed that during the transportation process, FVs were highly correlated to the network size of a city and demonstrated agglomeration characteristics only in the county-level cities [11]. Puente-Mejia et al. (2020) proposed a model based on observation and declarative data collection and discussed the method of combining observation data with declaration data to describe freight generation. Finally, it was found that the model could significantly increase the mobile understanding and network connectivity of FVs [12].

During the operation of the IoV, the collaborative communication between Vehicle to Roadside (V2R) and Vehicle to Vehicle (V2V) greatly increases the communication capabilities of the IoV. However, the optimization of its ND is also extremely important, which have been explored by many researchers. Contreras-Castillo et al. (2017) discussed the benefits of the IoV and the latest-formulated industry standards, thereby promoting the implementation of the IoV in the context of the increasing number of Internet-connected vehicles and the constantly updated vehicle network requirements. Finally, a communication protocol was proposed for the seamless integration and operation of the IoT [13]. Wang et al. (2018) proposed a feasible solution to enable real-time traffic management in the fog-based Internet of Vehicle system, thereby enabling offloading to minimize the average response time of vehicle reported events. In addition, an approach to solving the optimization problem of unloading was proposed. The performance of the actual taxi trajectory dataset was analyzed to prove the superiority of the method [14]. For the security of IoV in data transmission, Chen et al. (2019) proposed an authentication protocol for the IoV. However, the protocol was found to be suffered from offline identity guessing attacks, location spoofing attacks, and replay attacks. Meanwhile, it cost a long authentication time. After making several improvements to these shortcomings, it was found that the security and various performances of the protocol were greatly improved [15]. Wang et al. (2020) introduced the agent to the offloading of computing tasks, proposed a new drone-assisted mobile edge computing (MEC) framework, and used the intelligence and perception of the agent to build a system model. The simulation showed that introducing the agent could significantly reduce the delay and energy consumption. Also, the effectiveness of the agent was explained [16].

The above results suggest that scholars from various countries have systematically researched IOV in detail. However, in summary, there are various studies on data extraction of FVs and connected vehicle systems. However, studies on ND optimization are rare. Also, effective and complete research results for the IoV network deployment have not been reported yet. Therefore, this study uses FG to build a freight ILP model. Then, this study explores its ND optimization in the Internet of Vehicle system, providing wider applications of FVs in the IoV ND.

## 3. Methods

### 3.1 FG

FG is a new concept based on cloud computing. As a virtualized network platform, it is often deployed at the edge of the network and provides a distributed computing model of localized network services for devices. The FG layer uses network equipment to provide computing, storage, and network communication services, which greatly improves the network broadband and response speed of the system. It can also continue to provide services through FG in areas without network connections [17]. The purpose of FG is to provide users with powerful computing and communication resources at the edge of the network that is close to the user. Then, it provides a localized and efficient connection service, which overcomes the shortcomings of long distance and long delay from users in cloud computing. Generally, FG can be divided into six layers, i.e., the physical resource layer, the monitoring layer, the pre-processing layer, the data temporary storage layer, the security layer, and the transmission layer, as shown in Fig 1 [18].

**Fig 1:** The hierarchy diagram of FG.

The physical resource layer is the lowest layer in the FG hierarchy. It contains many equipment clusters and servers that support FG. It can manage and maintain physical nodes, wireless networks, virtual nodes, and virtual sensors in the environment, as well as integrate resources to provide infrastructure services to upper layers in the form of virtual resources. The monitoring layer is the most important layer in the FG hierarchy. It is mainly responsible for tasks such as reasonable allocation of resources in FG nodes, detection or recovery of node failures, detection and recording of FG underlying nodes and network activity status, and resource usage. It is also responsible for monitoring the energy consumption of equipment or nodes in FG, which provides data support. The pre-processing layer is mainly used for data management, which collects data for filtering, processing, and reconstruction. The temporary storage layer is mainly used to temporarily store the data obtained by the preprocessing layer. After the data are transferred to the cloud, the layer will delete the corresponding data backup from the local storage. The security layer is responsible for the security management of fog services in each layer, which achieves the full protection of data and resources and ensures the confidentiality of data. The transport layer is responsible for sending data obtained by the processing to the cloud; thus, the burden on the network core is minimized; ultimately, it provides more services as a platform.

### 3.2 IoV

The ND of connected vehicles usually requires rich connection methods and interactions. For current urban traffic monitoring systems, the communication technology used by the camera to the local data center is often multi-hop, and some data that needs to be processed in real-time will appear. To a certain degree of network delay, FG requires less data transmission volume, has the ability to quickly process real-time data, improves local storage and computing capabilities, and eliminates bottlenecks in data transmission. Software-defined network (SDN), as a new type of network architecture, mainly separates the control plane from the data plane, and finally, realizes flexible control of network traffic [19]. Combining SDN with FG can effectively solve intermittent connections and high packet loss rates in the IoV, as well as optimizing and improving network deployment of the IoV through communication and consistent control between facilities. The network architecture of the IoV is similar to the IoT, as shown in Fig 2.

**Fig 2:** System and architecture of IoV.

In the architecture of the IoV, the perception layer mainly collects sensor information from vehicle nodes in the network and surrounding traffic and uses the ad hoc network of the vehicle to transmit data, thereby providing the most original and comprehensive application layer for the IoV. The information layer is mainly to connect the car network to the network, to ensure the reliable transmission of data through protocol conversion, and finally, to achieve remote public office and remote car networking. The application layer mainly includes the data service center and human-computer interaction interface. Through the processing of the data on the IoV, the basic functions of traffic information release, vehicle safety control, and human-computer interaction are finally realized, and real-time interaction and mass storage of information can be completed [20]. Therefore, compared with the traditional mobile Internet, the network of connected vehicles presents a dynamic topology, heterogeneous communication modes, diversified application types and service requirements, and small delays and high reliability required for road safety applications. In the traffic system, vehicles and road side units (RSUs) have corresponding coordinates. The speed of the vehicle x is defined as v, the driving path of the vehicle is L, the range of the RSU is a circle with a radius of R, and C is the boundary of the RSU coverage area; thus, L is a tangent to the circle within the RSU range [21]. Representing the vehicle travel path as the sum of the current position and the path that continues to travel, the path trajectory is:

$$L:f(t)=P_{current}+vt$$ (1)

Where: *P*_*current*_ represents the current position, the position of RSU in the coordinate system is (*C*_*x*_, *C*_*y*_), and its communication range is expressed as:

$$C:{\left(x-C_{x}\right)}^{2}+{\left(y-C_{y}\right)}^{2}=R$$ (2)

The two equations above are combined to obtain the following equation:

$${\left(P_{current}+vt-C_{x}\right)}^{2}\text{+}{\left(P_{current}+vt-C_{y}\right)}^{2}\;=R^{2}$$ (3)

The time node when vehicles entering RSU coverage range is assumed as t1, and the time node when vehicles leaving RSU coverage range is assumed as t2. Then, the position coordinate at each time node is expressed as follows:

$$P_{enter}=(P_{current}^{x}+v_{x}t_{1},P_{current}^{y}+v_{y}t_{1})$$ (4)

$$P_{leave}=(P_{current}^{x}+v_{x}t_{2},P_{current}^{y}+v_{y}t_{2})$$ (5)

The distance that vehicles drive within the RSU coverage range is shown in the following equation:

$$\begin{array}{c} d_{v2r}=∥P_{enter}-P_{leave}∥\\ =\sqrt{{\left(v_{cx}\times (t_{2}-t_{1})\right)}^{2}+{\left(v_{cy}\times (t_{2}-t_{1})\right)}^{2}} \end{array}$$ (6)

In actual life, the communication connection time for oncoming vehicles is usually short, and the communication radius of the on-board unit is often discussed in three cases. If *ν*_*a*_ > *ν*_*b*_, the communication connection time is:

$$t(a,b)=\frac{\frac{1}{2}d_{v2v}+d_{ab}}{v_{a}-v_{b}}$$ (7)

$$\frac{1}{2}d_{v2v}=r_{c}+d_{ab}$$ (8)

Where: *d*_*ab*_ is the relative distance between vehicle x and vehicle y, *r*_*c*_ is the communication range of vehicles, $\frac{1}{2}d_{v2v}$ is the sum of relative distance between vehicles and the communication range of vehicles. If *ν*_*a*_ < *ν*_*b*_, the communication connection time is:

$$t(a,b)=\frac{\frac{1}{2}d_{v2v}+d_{ab}}{v_{b}-v_{a}}$$ (9)

If *ν*_*a*_ = *ν*_*b*_, the speeds of two vehicles are the same, and the communication connection time is:

t(a,b)→∞ (10)

However, to ensure the quality and stability of data transmission on the Internet of Vehicle system and avoid generating more hops, it is necessary to find a communication path to ensure the longest communication connection time from the source node to the destination node, thereby optimizing the deployment of the Internet of Vehicle system.

### 3.3 Construction of freight ILP model based on FG

ILP is often used to solve network deployment problems. By establishing a mathematical model, network deployment problems are converted into mathematical problems, and optimal solutions are obtained by solving linear programming equations [22]. In this study, to monitor the traffic situation of FVs, FG and ILP are applied to FVs, and a freight ILP model based on FG is constructed, as shown in Fig 3.

**Fig 3:** ND of FG-based freight ILP model.

In this model system, taking the urban road environment as the application scenario, it consists of FV test points, RSU, FG units, and cloud computing centers. The FVs are connected to the RSU deployed on the roadside by using a wireless network. The RSU transmits the collected information to a nearby computing unit, and the FG unit calculates and transfers the collected information to a cloud server for permanent storage. As for the network deployment of this model, compared with the traditional cloud computing network architecture, the freight model under FG has more features. The first is that the network has low latency and high bandwidth. Second, the network is load-balanced. A large amount of data processing and calculations need to be completed by the server. The best access point and service path are considered as much as possible to ensure the quality and speed of data transmission for large-scale network deployment on the IoV. Finally, the network has low costs. On the premise of ensuring network performance, the total costs of network deployment and planning need to be controlled.

### 3.4 Simulations

The freight vehicles involved are small vehicles that are allowed to pass in the city during normal hours. Besides, these vehicles only travel among cities. To verify the model proposed in this study, a simulation experiment is performed by using the Matlab platform. The entire network scenarios are set. Considering the real conditions of city streets, the Manhattan distance is used to represent the distance between two nodes, which is represented by a straight-line connection between the two points. Manhattan distance is also called taxi distance, which is used to indicate the total absolute wheelbase of two points in the standard coordinate system. The equation is as follows:

$$c=|x_{1}-x_{2}|+|y_{1}-y_{2}|$$ (11)

To solve the problem of ND resources, according to the different traffic volume and business volume of FVs in different urban areas, three kinds of network scenario needs are proposed. In terms of the costs of ND, the normalized standard cost unit gcu is used. The network simulation parameters and different scale scenario configurations are shown in Tables 1 and 2.

**Table 1:** Parameter settings for network simulation.

Parameters	Values
Γ (Maximum coverage radius of RSU)	400 m
μ (The maximum capacity of TP that can be covered by RSU)	50
K (Number of types of fog equipment in different configurations)	4
L_max_ (Maximum communication distance between fog equipment and RSU)	1.2 km

**Table 2:** Configuration of scenarios with different scales.

Scenarios with different scales	Scenario A	Scenario B	Scenario C
Number of candidate gateway nodes (Gw)	2	3	5
Number of candidate fog nodes (Fog)	3	7	14
Number of candidate RSU nodes	10	20	40
Number of FVs	30	50	80

The steps for simulation are as follows:

1. Network scenarios and parameters are initialized, mainly including the selection of network-deployed scenarios. The candidate points and all parameters are set.
2. The wireless coverage is realized where the RSU and the vehicle test point coincide. The distance between each node is calculated and saved in the distance matrix. For each vehicle test point, under the condition of meeting the capacity limit, the nearest RSU node is chosen to connect through the algorithm and form a group with each RSU as the headset.
3. The RSU coverage nodes are re-allocated.
4. A directed acyclic graph of the network is generated.

According to the number of RSU nodes connected to the fog equipment, different configurations are selected, and the costs of different sets are calculated, respectively. The minimum value is selected as the minimum cost of network deployment. The running time is recorded during operation.

## 4. Results and discussion

### 4.1 Analysis of ND results of different scenarios

For the analysis of network deployment in different scenarios, the results obtained are shown in Figs 4–6. The horizontal and vertical coordinates here have no practical meanings; they are only to simplify the city streets into a 20*20 area. As shown in the figures, the RSU utilization is the highest in Scenario A, and a higher proportion of monitoring of FVs is possible. As the scale of the scenario continues to increase, such as Scenario B and Scenario C, the network complexity gradually increases and the solution time is obvious increasing, thereby greatly reducing the operating efficiency. Therefore, the freight ILP model based on fog calculation is more suitable for small-scale scenarios, i.e., Scenario A can optimize the objective function, and the utilization rate is low in large-scale scenarios.

**Fig 4:** ND analysis of Scenario A.

**Fig 5:** ND analysis of Scenario B.

**Fig 6:** ND analysis of Scenario C.

### 4.2 Analysis of network costs and running time of different scenarios

When analyzing the network cost and computing time of different scenarios, the FG of this study is compared with the traditional cloud computing solution. The results are shown in Figs 7 and 8. As shown in Fig 7, in the analysis of operating costs, the difference between FG and traditional cloud computing solutions in different scenarios is not obvious, and the cost of FG is slightly lower. Furthermore, by observing the running time of the two groups of solutions, it is found that in network Scenario C, the running time of traditional cloud computing solutions increases exponentially, while the running time of FG has not changed significantly. Therefore, as can be inferred from the comparison of network costs and running time, the network deployment solution based on FG requires less costs, shorter running time, and has apparent effectiveness and efficiency.

**Fig 7:** Comparative analysis of network costs of different schemes under each scenario.

**Fig 8:** Comparative analysis of running time of different schemes under each scenario.

Fog computing and traditional methods are utilized respectively to solve different network scenarios. The obtained total cost is not much different; however, their running time is significantly different. With the continuous expansion of network scenarios, the running time of traditional methods gradually increases exponentially; sometimes, the scenario even cannot be solved. However, the running time of the fog computing method is only a few seconds, which can be controlled in a small range in different scenarios. Therefore, the method of fog computing is more efficient.

The specific optimization results of the two algorithms, i.e., the traditional method and the fog computing method, are shown in Table 3:

**Table 3:** Detailed comparison results of different methods in various scenarios.

Scenarios	Scenario 1		Scenario 2		Scenario 3	
Methods	Traditional	Fog computing	Traditional	Fog computing	Traditional	Fog computing
Running time (s)	19.42	0.172	2037	0.374	5842	0.410
Network total cost (gcu)	53410	58942	63121	69748	94031	10357
Difference in cost	8.13%		12.2%		9.6%	

## 5. Conclusions

A freight-ILP model based on FG is built, and the application of ND optimization in the network-to-vehicle system is explored through this model through simulation. The results show that the proposed model is more suitable for small-scale scenarios and can optimize the objective function; however, its utilization rate is low in large-scale scenarios. Compared with traditional cloud computing solutions, the ND solution based on FG requires less cost, shorter running time, and has apparent effectiveness and efficiency.

In summary, the FG-based freight ILP model constructed in this study is more suitable for small-scale scenarios. Meanwhile, the model has a short running time, requires less cost, and has apparent effectiveness and efficiency, providing experimental evidence for the optimization of FV ND in the IoT system. However, deficiencies also exist in this study. For example, this study mainly simulates the real vehicle networking environment through relevant simulation experiments. However, other complex factors need to be considered in the actual large-scale network deployment. Therefore, in the subsequent study, field inspections will be conducted to make the deployment closer to the actual network environment, thereby making the results more practical. Due to the time limitations, the results have not been applied in reality. Therefore, in the future, applying the research results practically and conducting tests are important research directions.

## Supporting information

S1 Data (XLS)
